The article "Correlation between High Myopia Susceptibility and Polymorphisms of RASGRF1 Gene among College Students in Zhejiang" was retracted in 2023. Reasons: signs of a paper mill; compromised peer review; unreliable results or conclusions; concerns about the peer review.

# Correlation between High Myopia Susceptibility and Polymorphisms of RASGRF1 Gene among College Students in Zhejiang

**DOI:** 10.1155/2023/6767410

**Published:** 2023-02-21

**Authors:** Jipan Yi, Yingying Dai, Shangsheng Ma, Yiyi Zheng, Yunjie Liang, Xiaojie Huang

**Affiliations:** Optometry Technology of Zhejiang Industry and Trade Vocational College, Wenzhou 325000, Zhejiang, China

## Abstract

**Objective:**

The aim of the study is to analyze the correlation between high myopia susceptibility and Ras protein-specific guanine nucleotide-releasing factor-1(RASGRF1) gene polymorphism among college students in Zhejiang.

**Methods:**

A stratified whole-group sampling method was used to select 218 cases of college students in Zhejiang who met the inclusion and exclusion criteria from January, 2019, to December, 2021, and they were divided into 77 cases (154 eyes) in the high myopia group and 141 cases (282 eyes) in the medium-low myopia group according to the degree of myopia, and 109 cases of college volunteers without myopia from the same period of medical examination in the region were included in the control group. The single nucleotide polymorphisms (SNPs) located in functional regions were selected by searching the literature and genetic databases, and the base sequences of rs939658, rs4778879, and rs8033417 loci were obtained by genotyping candidate SNPs using multiplex ligase detection reaction technique. The cardinality test was used to compare the differences in genotype frequency distribution of each locus of the RASGRF1 gene between the high myopia group and the low to moderate myopia group and the control group.

**Results:**

The genotype frequencies and allele frequencies of the RASGRF1 gene rs939658 locus in the high myopia group compared with the moderate-low myopia group and the control group were not statistically significant (*P* > 0.05). The genotype frequencies and allele frequencies of the rs4778879 locus of the RASGRF1 gene were compared among the three groups, and the differences were not statistically significant (*P* > 0.05). The genotype frequency and allele frequency of the rs8033417 locus of the RASGRF1 gene differed significantly among the three groups (*P* < 0.05).

**Conclusion:**

The polymorphism of the rs8033417 locus of the RASGRF1 gene was significantly correlated with the susceptibility of high myopia among college students in Zhejiang.

## 1. Introduction

High myopia refers to pathological myopia with a refractive error of -6D and above; its main symptoms are progressive vision loss and, in severe cases, irreversible pathological changes that cannot be optically corrected, such as chorioretinal degeneration, glaucoma, cataract, and retinal detachment [1, 2]. Some studies have found that the prevalence of high myopia among college students in China has shown a significant upward trend in recent years, which has a negative impact on their quality of life and employment [3, 4]. The formation of high myopia is more genetically related, and the latest human genetic library data show that hundreds of genetic factors associated with myopia have been determined by genome-wide association studies and whole-exome sequencing [5], among which Ras protein-specific guanine nucleotide-releasing factor 1 (RASGRF1) is a gene closely associated with myopia as confirmed by several studies [6]. RASGRF1, located on chromosome 15, is highly expressed in the retina and optic neurons and is important for eye development and visual signaling; mutations in this gene can activate Ras, causing overgrowth of the eye and leading to the development of high myopia [7]. Kim and Baek [8] showed that the association studies and linkage analysis of RASGRF1 gene polymorphisms with high myopia varied widely in different populations, so the association of RASGRF1 gene with myopia needs to be further validated in different populations. Based on this, this study was conducted to analyze the association between high myopia susceptibility and RASGRF1 gene polymorphism among college students in Zhejiang, with the aim of further clarifying whether RASGRF1 gene is an important pathogenic gene affecting the occurrence of high myopia among college students in this region.

## 2. Materials and Methods

### 2.1. General Information

A stratified whole-group sampling method was used to randomly select three universities from the Zhejiang region from January, 2019, to December, 2021, and all freshman students within five classes from each university who volunteered to participate in this study were randomly selected. A total of 529 college students voluntarily participated in this study, and 218 cases finally met the inclusion and exclusion criteria, including 121 males and 97 females, with an average age of (20.86 ± 3.47) years.

Inclusion criteria were as follows: aged 18–24 years old; Han nationality; met the diagnostic criteria for myopia [9]; all had binocular onset; no strabismus or amblyopia; no history of ocular trauma or surgery; and patients and their families understood and gave informed consent.

Exclusion criteria were as follows: combined with severe heart, liver, kidney, and other organ dysfunction and other immune-related diseases; combined with systemic acute and chronic diseases affecting vision such as diabetes; combined with glaucoma, cataract, retinal, or optic neuropathy; and combined with malignant tumor or psycho-psychiatric diseases. They were divided into 77 cases (154 eyes) in the high myopia group and 141 cases (282 eyes) in the medium-low myopia group according to the myopia grading standard, and 109 college volunteers without myopia from the same period of medical examination in Zhejiang were included in the control group. Myopia grading standard [10]: high myopia was determined by the equivalent spherical lens of both eyes ≥−8.0 D and the axis length (AL) ≥26 mm; low-moderate myopia was determined by the equivalent spherical lens of both eyes −0.5 D to −7.75 D.

### 2.2. Methods

#### 2.2.1. Routine Ophthalmic Examination

All study subjects underwent routine ophthalmic examinations and special instrumental examinations, including ① naked distance and near visual acuity and corrected visual acuity in both eyes. ② Topcon RM8800 computerized optometry was used for binocular computerized optometry, and Topcon comprehensive optometry was used for binocular dilated optometry and trial lenses to check refractive status, determine refractive error, and calculate spherical equivalent (SE). ③ Using Topcon NCT CT-80 tonometer, the intraocular pressure of both eyes was detected. ④ The corneal status, anterior chamber depth, pupil size and shape, and crystal transparency were observed by slit-lamp microscope Topcon SL-1E. ④ After the pupil was dilated fully with the front lens, fundus examination was performed with the front lens under the slit lamp, focusing on the macular area. ⑤ The eye movements of both eyes were examined. ⑥ AL was examined in both eyes using a diagnostic A-ultrasound machine, and each eye was measured three times to obtain the mean value for analysis.

#### 2.2.2. RASGRF1 Gene SNP Selection

By searching the literature and gene databases, single nucleotide polymorphisms (SNPs) located in functional regions were selected, and loci with disease susceptibility were selected in combination with the literature, and the minimum allele frequency (MAF) of SNP was screened, and SNP loci with MAF > 10% were selected for function prediction, with priority given to loci with larger MAF values. RASGRF1 and its upstream 100 kb range of ccRE sequences were screened from the gene database, and two SNPs were finally selected for genotyping analysis in combination with existing literature studies. There were 5 inheritance patterns, namely, allelic model (A_1_ vs A_2_), homozygous model (A_1_ A_1_ vs A_2_A_2_), heterozygous model (A_1_ A_1_ vs A_1_A_2_), dominant model (A_1_ A_1_ + A_1_ A_2_ vs A_2_A_2_), and implicit model (A_2_A_2_ vs A_1_ A_2_ + A_2_ A_2_).

#### 2.2.3. SNP Genotyping and Sequencing

SNP typing was performed using a modified multiplex ligase detection reaction (LDR) technique with polymerase chain reaction (PCR) primers designed using Primer3v.0.4.0 and synthesized by Dalian Baocheng Biological Company. Primer sequences: rs939658 Forward 5′-CCACGCAGCATTCATTCACTTG-3′ and Reverse 5′-CCTCCCCTCATGGGTACCTGTC-3′; rs4778879 Forward 5′-GAAACTGGGCAGGCTGAGAACA-3′ and Reverse 5′-GCTGGTATTCCAAAACTCCATGTAGAA-3′; and rs8033417 Forward 5′ -TGGAGCAGCTGGGGATGGGG-3′ and reverse 5′-AGCCGAGATGACACCACTGCA-3′. The ABI3730XL sequencer from Applied Biosystems was used to perform the assay, and the typing data were analyzed using GeneMapper software. The typing process ensured that the negative control was band-free, and in addition, 10% of the samples were randomly selected for sequencing and validation of replicate experiments to ensure the reliability of the assay results.

### 2.3. Statistical Processing

SPSS 22.0 statistical software was used for data analysis, and the Hardy–Weinberg equilibrium test of the genotypes of each SNPs locus in the high myopia group and the control group and the moderate-low myopia group was used to determine the population representativeness of the samples by the *χ*^2^ test. Measurement data were expressed by $\left(\bar{x}\pm s\right)$ and the differences between groups were expressed by two-sample independent *t*-test; the count data were expressed as rate and the differences between groups were expressed by *χ*^2^ test; the difference was considered statistically significant by two-sided *P*  <  0.05.

## 3. Results

### 3.1. Basic Situation

This study included 218 college students in Zhejiang, of which female students were more common, accounting for 59.74%. The grouping according to the degree of myopia could be divided into 77 cases (154 eyes) in the high myopia group and 141 cases (282 eyes) in the low to moderate myopia group, and 109 college students with eyes without myopia were selected as a normal control group. Statistical analysis of age (Figure 1(b)) and gender (Figure 1(a)) among the three groups showed that there was no statistically significant difference between the three groups in the abovementioned aspects of comparison (*P* > 0.05); the axial length (Figure 1(c)) and SE (Figure 1(d)) of each group were different (*P* < 0.05). As shown in Figure 1.

### 3.2. Hardy–Weinberg Equilibrium Test and Distribution of RASGRF1 Gene SNP Loci

The results of the H–W balance test showed that the genotype distribution of SNP loci in the high myopia group, low to moderate myopia group, and control group were not statistically significant (*P*  >  0.05) compared with the distribution in the H-W theoretical state. It indicated that the distribution of genotypes in the high myopia group, moderate-low myopia group, and control group had reached a genetic balance, and the population was representative, and further analysis could be carried out as shown in Table 1.

### 3.3. Comparison of Genotype Distribution and Allele Frequency of the rs939658 Locus of RASGRF1 Gene among Three Groups

The genotype frequencies and allele frequencies of the rs939658 locus of the RASGRF1 gene in the high myopia group compared with the low-moderate myopia group and the control group were not statistically significant. (*P* > 0.05), as shown in Table 2.

### 3.4. Comparison of Genotype Distribution and Allele Frequency of RASGRF1 Gene rs4778879 Locus among Three Groups

The genotype frequencies and allele frequencies of the RASGRF1 gene rs4778879 locus in the high myopia group compared with the low-moderate myopia group and the control group were not statistically significant (*P* > 0.05), as shown in Table 3.

### 3.5. Comparison of Genotype Distribution and Allele Frequency of RASGRF1 Gene rs8033417 Locus among Three Groups

The genotype frequency and allele frequency of the rs8033417 locus of the RASGRF1 gene in the high myopia group compared with the low to moderate myopia group and the control group were statistically significant (*P* < 0.05), as shown in Table 4.

## 4. Discussion

High myopia is an eye disease caused by the interaction of genetic, environmental, and individual differences. In China, the prevalence of high myopia among college-level students accounts for about 20% of the number of myopic college students, and the accompanying complications such as chorioretinopathy and glaucoma are common causes of vision loss and even blindness in the naked eyes of adolescents [10, 11]. With the application of molecular genetics and genotyping technology in clinical medical research, the study of genetic susceptibility and pathogenesis of myopia has entered a new phase of exploration. The application of molecular genetic methods to study and analyze the genetic factors and susceptibility genes of high myopia provides a molecular genetic basis for clinical development of high myopia prevention and treatment programs [12]. Various gene sequence-mediated signaling pathways have been found to be involved in the development of myopia, among which genetic variants at the RASGRF1 locus have been associated with visual function and several of its SNP loci may be closely associated with high myopia [13], but analysis of the correlation between RASGRF1 gene polymorphisms and susceptibility to high myopia has been less frequently reported.

This study considered college students in Zhejiang as the research subject and screened out the genes by searching the relevant literature in NCBI PubMed; we screened the genes and SNP loci that might be associated with high myopia and finally identified rs939658, rs4778879, and rs8033417 loci on RASGRF1 gene, and analyzed their relationship with the susceptibility to high myopia of college students in this region. The Hardy–Weinberg equilibrium test showed that the genotype distributions of SNP loci in the three groups were not significantly different from those in the H–W theory state, indicating that the genotype distributions in all three groups reached genetic equilibrium and the populations were representative. In this study, the genotype frequency and allele frequency of SNP rs939658 and rs4778879 of the RASGRF1 gene between the myopia group and the control group were not significantly different, but the genotype frequencies and allele frequencies of the rs8033417 locus of the RASGRF1 gene were significantly different between the two groups, in which the risk of high myopia was significantly higher in C allele carriers than in T allele carriers, indicating that the C allele of the rs8033417 locus was associated with myopia. The RASGRF1 gene, a protein-coding gene localized at 15q25.1, is highly expressed in neurons and the retina, and its expression is regulated by retinol and muscarinic receptors and plays an important role in retinal function and enhanced visual process [14, 15]. Defects in the RASGRF1 gene cause impaired regulation of retinol and muscarinic receptors, resulting in impaired visual development and increased risk of high myopia [16, 17]. Kunceviciene et al. [18] found that the RASGRF1 gene was associated with the heritability of myopia, in which the rs8027411GT type carriers were 2.7-fold more likely to develop myopia, similar to the results of the present study, suggesting that the focus should be on the rs8033417 locus C carriers and timely and effective preventive measures should be given to slow down the development of myopia.

In this study, we further analyzed the genotype distribution and allele frequency of RASGRF1 gene polymorphism SNP loci in patients with different degrees of myopia, and the results showed that there was no significant difference in the genotype and allele frequencies of SNPs rs939658 and rs4778879 in the RASGRF1 gene in the high myopia group and low to moderate myopia group, while the genotype frequencies and allele frequencies of rs8033417 loci of RASGRF1 gene in both groups were significantly different. This suggests that the genetic susceptibility to high myopia among college students in Zhejiang is not significantly associated with the rs939658 and rs4778879 loci of the RASGRF1 gene, while the rs8033417 locus may be a risk gene for high myopia among college students in this region while carrying the C allele, and college students carrying the C allele have an increased risk of myopia. However, no evidence was found in the study of Fernandez-Medarde and Santos [19] to support the association of high myopia with the rs8033417 locus of the RASGRF1 gene, and analysis of the reasons for this may be related to the different single nucleotide polymorphism loci selected in this study, and differences in the inclusion criteria for high myopia can also cause changes in gene frequency [20]. The study of SNPs and genetic susceptibility of specific myopia groups is important for understanding the molecular genetic mechanisms underlying the development of high myopia in different populations in various regions. The disadvantage of this study is that the number of samples selected is relatively limited, and the included research subjects are all Han college students in the region. Considering that high myopia is a complex process involving multiple genes and pathways, the subsequent experimental validation of the function of the rs8033417 locus of the RASGRF1 gene is still needed to increase the sample size [21].

In conclusion, this study confirmed that the high myopia susceptibility of college students in Zhejiang was associated with the rs8033417 locus of the RASGRF1 gene and that college students carrying the C allele were at increased risk of myopia. In this study, we identified the rs8033417 locus variation in the RASGRF1 gene in a population of college students with high myopia in Zhejiang, which provided a reliable molecular genetic basis for the later gene diagnosis and treatment and prevention of high myopia for college students in the region.

## Figures and Tables

**Figure 1:** Demographic characteristics among the three groups.

**Table 1:** Hardy–Weinberg equilibrium test for SNP loci of RASGRF1 gene.

SNP ID	*High myopia group (n* *=* *77)*		*Moderate-low myopia group (n* *=* *141)*		*Control group (n* *=* *109)*	
	A_1_A_1_/A_1_A_2_/A_2_A_2_	*P*	A_1_A_1_/A_1_A_2_/A_2_A_2_	*P*	A_1_A_1_/A_1_A_2_/A_2_A_2_	*P*
rs 939658	21/15/41	0.257	44/23/74	0.386	34/26/49	0.163
rs 4778879	17/22/38	0.581	25/43/73	0.356	24/39/46	0.465
rs 8033417	12/16/49	0.096	32/67/42	0.065	23/47/39	0.291

A_1_ means mutant type, A_2_ means wild type, A_1_A_1_ means mutant homozygous type, A_1_A_2_ means heterozygous genotype, and A_2_A_2_ means wild type homozygous type.

**Table 2:** Comparison of genotype distribution and allele frequency of the rs939658 locus of RASGRF1 gene among three groups.

Genotype/alleles		High myopia group (*n* = 77)	Moderate-low myopia group (*n* = 141)	Control group (*n* = 109)	*χ* ^2^	*P*
Genotype	GG	21	44	34	2.974	0.562
	GA	15	23	26		
	AA	41	74	49		

Alleles	G	57	111	94	1.502	0.472
	A	97	171	124		

**Table 3:** Comparison of genotype distribution and allele frequency of RASGRF1 gene rs4778879 locus among three groups.

Genotype/alleles		High myopia group (*n* = 77)	Moderate-low myopia group (*n* = 141)	Control group (*n* = 109)	*χ* ^2^	*P*
Genotype	GG	17	25	24	2.820	0.588
	GA	22	43	39		
	AA	38	73	46		

Alleles	G	56	93	87	2.567	0.277
	A	98	189	131		

**Table 4:** Comparison of genotype distribution and allele frequency of RASGRF1 gene rs8033417 locus among three groups.

Genotype/alleles		High myopia group (*n* = 77)	Moderate-low myopia group (*n* = 141)	Control group (*n* = 109)	*χ* ^2^	*P*
Genotype	TT	12	32	23	25.684	<0.001
	CT	16	67	47		
	CC	49	42	39		

Alleles	T	40	131	93	18.070	<0.001
	C	114	151	125		

## Data Availability

The data used and/or analyzed during the current study are available from the corresponding author on reasonable request.
